The article "Exploiting Feature Selection and Neural Network Techniques for Identification of Focal and Nonfocal EEG Signals in TQWT Domain" was published in 2021. Journal: J Healthc Eng.

# Exploiting Feature Selection and Neural Network Techniques for Identification of Focal and Nonfocal EEG Signals in TQWT Domain

**DOI:** 10.1155/2021/6283900

**Published:** 2021-08-27

**Authors:** Muhammad Tariq Sadiq, Hesam Akbari, Ateeq Ur Rehman, Zuhaib Nishtar, Bilal Masood, Mahdieh Ghazvini, Jingwei Too, Nastaran Hamedi, Mohammed K. A. Kaabar

**Affiliations:** ^1^Department of Electrical Engineering, The University of Lahore, Lahore 54000, Pakistan; ^2^Department of Biomedical Engineering, South Tehran Branch, Islamic Azad University, Tehran, Iran; ^3^Department of Electrical Engineering, Government College University, Lahore 54000, Pakistan; ^4^Department of Electrical Engineering, Superior University, Lahore 54000, Pakistan; ^5^School of Electrical Engineering, Xi'an Jiaotong University, Xi'an 710049, China; ^6^Department of Computer Engineering, Faculty of Engineering, Shahid Bahonar University of Kerman, Kerman, Iran; ^7^Faculty of Electrical Engineering, Universiti Teknikal Malaysia Melaka, Malacca, Malaysia; ^8^Department of Biomedical Engineering, Faculty of Electrical Engineering, K. N. Toosi University of Technology, Tehran, Iran; ^9^Gofa Camp,Near Gofa Industrial College and German Adebabay, Nifas Silk-Lafto, Addis Ababa 26649, Ethiopia; ^10^Jabalia Camp,United Nations Relief and Works Agency (UNRWA), Palestinian Refugee Camp, Gaza Strip, Jabalya, State of Palestine; ^11^Institute of Mathematical Sciences, Faculty of Science, University of Malaya, Kuala Lumpur 50603, Malaysia

## Abstract

For drug resistance patients, removal of a portion of the brain as a cause of epileptic seizures is a surgical remedy. However, before surgery, the detailed analysis of the epilepsy localization area is an essential and logical step. The Electroencephalogram (EEG) signals from these areas are distinct and are referred to as focal, while the EEG signals from other normal areas are known as nonfocal. The visual inspection of multiple channels for detecting the focal EEG signal is time-consuming and prone to human error. To address this challenge, we propose a novel method based on differential operator and Tunable Q-factor wavelet transform (TQWT) to distinguish the focal and nonfocal signals. For this purpose, first, the EEG signal was differenced and then decomposed by TQWT. Second, several entropy-based features were derived from the TQWT subbands. Third, the efficacy of the six binary feature selection algorithms, binary bat algorithm (BBA), binary differential evolution (BDE) algorithm, firefly algorithm (FA), genetic algorithm (GA), grey wolf optimization (GWO), and particle swarm optimization (PSO), was evaluated. In the end, the selected features were fed to several machine learning and neural network classifiers. We observed that the PSO with neural networks provides an effective solution for the application of focal EEG signal detection. The proposed framework resulted in an average classification accuracy of 97.68%, a sensitivity of 97.26%, and a specificity of 98.11% in a tenfold cross-validation strategy, which is higher than the state of the art used in the public Bern-Barcelona EEG database.

## 1. Introduction

### 1.1. Background

Epilepsy is a disease of the central nervous system in which the brain is abnormally active [1–3]. Epilepsy, in other words, is a neurological disorder that causes seizures, abnormal sensations, and sometimes loss of consciousness [4]. Epilepsy patients experience recurrent seizures due to elevated electrical activity in the brain, which disrupts the connection between the brain synapses. Although seizure symptoms might affect any part of the body, electrical disorders related to all of them occur in the brain. The biggest challenge in neuroscience is understanding the behavior of epilepsy and its effect on the brain. Determining the type of seizure, the location of the attack, how it spreads, the amount of brain that is affected, and how long it lasts plays an important role.

Around 50 million of the world's population, most of whom living in developing countries, suffer from epilepsy [5]. Neurologists classify epilepsy into two categories, partial or focal and generalized epilepsy. If epilepsy attachments occur in limited areas of the brain, this is called focal epilepsy, and if the whole brain is involved, this is called general seizure (see Figure 1).

Epilepsy can afflict anyone at any age, but it can be cured by using antiepilepsy medications. The results of the antiepilepsy drugs are promising, but 25% of patients do not respond well to antiepilepsy drugs [6]. 20% of patients with generalized epilepsy and 60% of patients with focal epilepsy are not treated by antiepilepsy drugs. Surgery is a treatment option for patients with focal epilepsy who are not responding well to antiepilepsy drugs. In such cases, a physician eliminates brain areas that are the source of the epilepsy attack. However, a significant step before surgery is to localize these areas of the brain. Although positron emission tomography (PET) scan [7], single-photon emission computed tomography (SPECT) scan [8], and magnetic resonance imaging (MRI) [9] can localize focal areas of the brain, the main problem is the inaccessibility of this equipment in most of the developing countries.

Electroencephalogram (EEG) signals measure the electrical activity of brain synapses. The EEG signals are commonly used by physicians to diagnose brain disorders or activities. The physician may localize the focal areas of the brain by visual inspection of the EEG signal. In focal epilepsy patients, EEG signals recorded from the focal areas of the brain are distinct and are known as the focal EEG signals. In contrast to focal signals, nonfocal signals are recorded from other parts of the brain (see Figure 1). Visual inspection of multiple channels for detecting the focal EEG signal is time-consuming and vulnerable to human error. Therefore, a computer diagnostic system is required for the accurate detection of focal signals.

### 1.2. Previous Works

Several machine learning methods have been developed in the literature based on linear and nonlinear features for the classification of focal and nonfocal EEG signals. Any machine learning method has three main steps: (1) feature extraction, (2) feature selection, and (3) classification. We can categorize previous works according to these three steps.

The linear and nonlinear features have been extracted from the EEG signal from the time domain, frequency domain, and time-frequency domain.

In [10] delay permutation entropy and in [11–13] a combination of linear and nonlinear features have been extracted from EEG signals in the time domain. In other words, these features have been extracted directly from EEG signals. The features extracted from the EEG signal spectrum are frequency-domain features such as [14] in which the EEG signal spectrum was computed by Fourier transform (FT) and mean frequency and root mean square were extracted as discrimination features.

Many time-frequency methods like empirical mode decomposition (EMD) [15–17], s-transform [18], discrete wavelet transform (DWT) [19–21], EMD-DWT [6], empirical wavelet transform (EWT) [22–24], flexible analytic wavelet transform (FAWT) [25, 26], Fourier-Bessel series expansion domain empirical wavelet transform filter bank (FBSE-EWT) [27], Fourier-Bessel series expansion based flexible time-frequency coverage wavelet transform (FBSE-fTF-cwt) [28], sliding mode-singular spectrum analysis (SM-SSA) [29], variational mode decomposition (VMD) [30], and VMD-DWT [31] have been used for decomposing EEG signals. Most of the extracted features from the time-frequency representation of EEG signals are entropy-based features that indicate appropriate entropies in the classification of focal and nonfocal EEG signals.

Sample entropy [15, 16], Shannon entropy [6, 16, 19], Renyi's entropy [6, 16, 19], approximate entropy [16], phase entropies [16, 19], log energy (LE) entropy [6, 17, 24–26, 32], Stein's unbiased risk estimate (SURE) entropy [17, 24, 25], Tsallis wavelet entropy [19], fuzzy entropy [19, 26, 31], and permutation entropy [19] have been extracted previously from EEG signals coefficients as discrimination feature for classification of focal and nonfocal EEG signals.

After extracting the features, the significant features must be selected and fed to classifiers. The feature selection is an important step for designing machine learning applications since if the number of features fed to the classifier is very high, the complexity of the system increases; on the contrary, if the number of features is very low, the accuracy (ACC) of the system decreases and the machine is unable to decide correctly. Almost all of the previously proposed machine learning methods in focal and nonfocal signal classification application use *p* value for selecting significant features [6, 11, 13, 14, 16, 17, 19, 22, 23, 25, 26, 31, 33–35], in such a way that features with *p* values less than 0.05 were significant and could be used as an input to classifiers. Although this traditional method can select significant features, it cannot be used as a significant feature selection tool when all of the extracted features have a *p* value less than 0.05. In this case, search heuristic approaches can be used as a feature selection method. In other words, these approaches optimize the number of feature vector arrays for resulting in the best classification performance. In this work, we used six binary optimization methods for selecting significant features, namely, binary bat algorithm (BBA), binary differential evolution (BDE) algorithm, firefly algorithm (FA), genetic algorithm (GA), grey wolf optimizer (GWO), and particle swarm optimization (PSO).

Support vector machine (SVM) and *K*-nearest neighbor (KNN) algorithms are two well-known classifiers used previously for the classification of focal and nonfocal EEG signals. Although the performance of these two algorithms for focal detection was acceptable, resulting in best classification performance, it is better to check the performance of the feed-forward neural network (FFNN), cascade-forward neural network (CFNN), generalized regression neural network (GRNN), and recurrent neural network (RNN) classifiers for focal detection application.

### 1.3. Contribution

EEG signal is nonstationary and complex [36–41]. Tunable Q-factor wavelet transform (TQWT) has been proposed for analyzing the nonstationary, nonlinear, and oscillatory signals [42].

Although TQWT was previously used for focal detection, the final results reported were not significantly proper [33] and involved intense calculations [34]. In this study, TQWT is used as a processing tool to decompose the focal and nonfocal EEG signals. The motivation stems from the successful deployment of TQWT in other biomedical signal processing applications such as detecting epileptic seizures [34, 43–49] and alcoholism [50] by EEG signals, detecting coronary artery disease [51] by heart rate variability (HRV) signals, heart valve [52, 53] and septal defects disorders [54, 55], aortic and mitral disorders [56, 57] by cardiac sound signals [58], detecting hand movements [59] and amyotrophic lateral sclerosis (ALS) disorder [60] by electromyogram (EMG) signals, and sleep apnea [61] by electrocardiogram (ECG) signals that indicate the ability of TQWT in biosignal processing application.

We can change the TQWT parameters to get optimal conditions that have resulted in the best classification performance. Recently, the authors showed the significant effect of differential operation in the classification of focal and nonfocal signals [23, 32]. Moreover, in previous studies, the results of entropy-based features were promising for both focal and nonfocal EEG classifications [6, 17, 33, 34]. For these reasons, the influence of entropy-based features on different EEG signals in the TQWT domain was focused on the present study. Therefore, the differences in EEG signal decomposed into several subbands using TQWT and entropy-based features including LE entropy, Log L2-norm (LL2) entropy, SURE entropy, and threshold (TH) entropy have been studied. In most of the previous works, Kruskal-Wallis statistical (KWS) test was used as a feature selection; but, in this work, various algorithms including BBA, BDE, FA, GA, GWO, and PSO are evaluated as feature selection techniques to reduce the number of input feature vector arrays which lead the classifier's calculation to be much simpler. Furthermore, the selected features are tested with six classifiers, KNN, SVM, FFNN, CFNN, GRNN, and RNN, classifiers in tenfold cross-validation strategy.

To the best of the authors' knowledge, the entropies of TQWT subbands of differenced EEG signals and BBA, BDE, FA, GA, GWO, and PSO algorithms as feature selection, as well as FFNN, CFNN, GRNN, and RNN classifiers, have not been previously employed for the focal and nonfocal EEG signals classification.

### 1.4. Organization

The paper is organized as follows: Section 2 explains the proposed method which consists of the description of the used databases, differential operator, TQWT, entropy-based features, feature selection, and classification algorithms. The results and discussion are presented in Sections 3 and 4, respectively. Finally, the conclusion of the article is represented in Section 5.

## 2. Proposed Method

In this study, TQWT extracts subbands of EEG signals after differencing and four entropy-based features are computed from subbands for discrimination between focal and nonfocal EEG signals. Feature vector arrays are reduced by feature selection techniques and fed to classifiers. The block diagram of the proposed method is shown in Figure 2.

### 2.1. Used Database

In this research, the Bern-Barcelona EEG dataset has been used for the evaluation of the proposed method [62]. The EEG signals of this dataset were recorded from five focal epilepsy patients who are candidates for brain surgery. This dataset consists of 3750 focal and 3750 nonfocal EEG signals. The sampling frequency was 512 and the duration of each signal is 20 seconds, so each signal has 10240 samples. Each signal has two columns, namely, “*X*” and “*Y*,” which have been recorded from adjacent channels. In this work, “*X*–*Y*” is used for noise reduction and interference effects [6, 17].  Figure 3 shows a sample of “*X*,” “*Y*,” and “*X*-*Y*” signals for focal and nonfocal groups. In this study, all signals containing more than 41.6 hours of EEG data in the Bern-Barcelona database are used.

### 2.2. Differential Operator

By assuming that *A*[*n*]=[*a*_1_, *a*_2_,…, *a*_*n*_] is a sequence with length *n*, the differential operator is defined as follows:

(1) $$\begin{array}{c} A_{\text{diffe}}=\left[a_{2}-a_{1},a_{3}-a_{2},\ldots ,a_{n}-a_{n-1}\right], \end{array}$$

where *A*_diffe_(*n*) denotes differential of *A* (*n*) with *n* − 1 samples.

### 2.3. Tunable Q-Factor Wavelet Transform

Tunable Q-factor wavelet transform has been proposed in [42] for analyzing complex and oscillatory signals like EEG. However, the traditional DWT is one of the most commonly used tools in signal analysis applications, but it has several defects including the fixed number of oscillations in the mother wavelet, the fixed oversampling rate, and the fixed bandwidths of the filter bank [61]. The TQWT is a proficient transform that overcomes the mentioned limitations for analyzing oscillatory signals by providing the tunability of the *Q*-factor [42]. The main input variables to this transform, which can be easily adjusted, include the number of decomposition levels denoted as (*J*), Q-factor represented as *Q*, and the total oversampling rate of *r*. *Q* represents the number of wavelet oscillations and *r* denotes the overlap between frequency responses. An increase in *Q* makes all frequency responses narrower, allowing more decomposition levels to span the same frequency range. An increase in *r* with a constant *Q* increases the degree of overlap between adjacent frequency responses, increasing the number of decomposition levels required for covering the same frequency range [59]. The low-pass and high-pass filters with *αf*_*s*_ and *βf*_*s*_ as the scaling parameters associated with the input signal *s* [*n*] having a sampling rate of  *f*_*s*_ and different decomposition levels are given as follows:

(2) $$\begin{array}{c} F_{0}\left(\omega \right)=\left\{\begin{array}{cc} 1, & \left|\omega \right|<\left(1-\beta \right)\pi ,\\ \theta \left(\frac{\omega +\left(\beta -1\right)\pi }{\alpha +\beta -1}\right), & \left(1-\beta \right)\pi \leq \left|\omega \right|<\alpha \pi ,\\ 0, & \alpha \pi \leq \left|\omega \right|\leq \pi , \end{array}\right)\\ F_{1}\left(\omega \right)=\left\{\begin{array}{cc} 0, & \left|\omega \right|<\left(1-\beta \right)\pi ,\\ \theta \left(\frac{\alpha \pi -\omega }{\alpha +\beta -1}\right), & \left(1-\beta \right)\pi \leq \left|\omega \right|<\alpha \pi ,\\ 1, & \alpha \pi \leq \left|\omega \right|\leq \pi , \end{array}\right) \end{array}$$

where *θ*(*ω*) represents the 2*π*-periodic power-complementary function selected as the frequency response of the Daubechies filter with two vanishing moments. Meanwhile,*θ*(*ω*) is defined by the following equation:

(3) $$\begin{array}{c} \theta \left(\omega \right)=0.5\left(1+\cos\left(\omega \right)\right){\left(2-\cos\left(\omega \right)\right)}^{1/2}\;\left|\omega \right|\leq \pi . \end{array}$$

A filter bank that was used to perform decomposition can also be used to reconstruct the original input signal with the selected subbands. *r* and *Q*-factor in terms of the parameters of the filter bank, that is, *α* and *β* [42], can be formulated as follows:

(4) $$\begin{array}{c} r=\frac{\beta }{1-\alpha },\\ Q=\frac{f_{c}}{BW}=\frac{2-\beta }{\beta }, \end{array}$$

where *f*_*c*_ and BW denote the center frequency and bandwidth of the subband *J*, respectively.

### 2.4. Entropy-Based Features

Nowadays, entropy is one of the most widely used tools in signal processing applications. In telecommunication, entropy measures the value of missed data, whereas, in physics, entropy matures the uncertainty or degree of disorder in a chaotic system. Generally, entropy can measure the complexity in a nonlinear system like the brain. In this study, LE entropy, LL2 entropy, SURE entropy, and TH entropy were extracted from EEG signal subbands as the discrimination feature between focal and nonfocal signals.

Let *S*[*n*]=[*s*_1_, *s*_2_, *s*_3_,…, *s*_*n*_] be the wavelet time series sequence corresponding to TQWT subbands.

Then, the LE [6, 17], LL2 [35], SURE [17, 24], and TH [17] entropies of *S*[*n*] can be defined as

(5) $$\begin{array}{c} \text{LL}2=\log\left(\overset{n}{\underset{i=1}{\sum }}{\left|s_{i}\right|}^{2}\right),\\ \text{LE}=\sum_{i=1}^{n}\log_{2}\left(s_{i}^{2}\right),\\ \text{SURE}=n-\#\left\{i\text{ such that }\left|s_{i}\right|\leq \varepsilon \right\}+\sum_{i=1}^{n}\min\left(s_{i}^{2},\varepsilon^{2}\right),\\ {\text{TH}}_{\text{En}}\left(s_{i}\right)=\left\{\begin{array}{cc} 1, & \left|S_{i}\right|>\varepsilon ,\\ 0, & \text{else where.} \end{array}\right)\; \end{array}$$

So,

(6) $$\begin{array}{c} {\text{TH}}_{\text{En}}=\;\#\left\{i\text{ such that }\left|s_{i}\right|>\varepsilon \right\}, \end{array}$$

where *s*_*i*_ and *ε* are the *i*^th^ represented samples of the signal and positive threshold, respectively. In this work, the value of *ε* is selected to be 0.2 in both SURE and TH entropies. Also, the entropy MATLAB function is used for the calculation of LE, LL2, SURE, and TH entropies. Thus, the entropy-based features can be extracted from the TQWT subbands.

### 2.5. Feature Selection

#### 2.5.1. Binary Bat Algorithm

A bat emits a sound and follows an echo that is reflected from the objects in the environment to prevent obstacles, discover prey, and locate their nests in the darkness [63]. Inspired by this behavior of bats, the bat algorithm was proposed. This algorithm uses artificial bats to find an optimal solution in an objective function. The binary bat algorithm (BBA) is a discrete version of the bat algorithm presented by Nakamura et al. [64]. In the BBA, the search space is limited to an n-dimensional Boolean hypercube, in which any bat may move at nodes and corners of the lattice. To select features, each feature is described by a binary bat position vector [63]. Therefore, the value of 0 indicates the absence of a feature, and the value of 1 indicates the presence of a feature. For a target function *f*(*x*), *x* = (*x*_1_,  *x*_2_,   …,  *x*_*n*_), the bat population starts with the position *x*_*i*_, velocity *v*_*i*_, and pulse frequency *f*_*i*_. Suppose that ${\hat{x}}^{j}$is the current global best solution in the dimension *j*, and *βϵ*[0,  1] is a random number. So, the velocity and position of the *i*th bat are updated as follows:

(7) $$\begin{array}{c} f_{i}=f_{\text{min}}+\left(f_{\text{min}}-f_{\text{max}}\right)\beta ,\\ v_{j}^{i}\left(t\right)=v_{j}^{i}\left(t-1\right)+{\hat{x}}^{j}-{\hat{x}}^{j}\left(t-1\right)f_{i},\\ x_{j}^{i}\left(t\right)=x_{j}^{i}\left(t-1\right)+v_{j}^{i}\left(t\right). \end{array}$$

At first, the pulse rate  *r*_*i*_, the loudness *A*_*i*_, and the maximum number of iterations *T* are initialized. Then, at each iteration, these parameters will be updated using the three following equations:

(8) $$\begin{array}{c} x_{\text{new}}=x_{\text{old}}+\varepsilon A\left(t\right), \end{array}$$

(9) $$\begin{array}{c} A_{i}\left(t+1\right)=\alpha A_{i}\left(t\right), \end{array}$$

(10) $$\begin{array}{c} r_{i}\left(t+1\right)=r_{i}\left(0\right)\left[1-e^{-\gamma t}\right], \end{array}$$

where we have variable *ε* *ϵ* [−1,  1] and *α*,  *β* are two constants. In each iteration, for each bat, the sigmoid function is applied using

(11) $$\begin{array}{c} S\left(v_{j}^{i}\right)=\frac{1}{1+e^{-v\left(i/j\right)}}, \end{array}$$

and the position is updated as follows:

(12) $$\begin{array}{c} x_{j}^{i}=\left\{\begin{array}{cc} 1, & \;if\rho \leq S\left(v_{j}^{i}\right),\\ 0, & \text{otherwise,} \end{array}\right) \end{array}$$

where *x*_*j*_^*i*^(*t*) and *v*_*j*_^*i*^(*t*) show the position and velocity of particle *i* at iteration *t* in dimension *j* and *ρ* ~ *U*(0,1). In our study, the BBA is iterated 40 times by using four bats and setting *α*= *β*=1.

#### 2.5.2. Differential Evolution Algorithm

The differential evolution algorithm is a heuristic population-based random search scheme for global optimization. Many objective functions are nondifferentiable, discrete, nonlinear, noisy, flat, multidimensional, constrained, or stochastic. Differential evolution algorithm can be exploited to solve such problems. Basic operations such as selection, crossover, and mutation are the basis of the difference algorithm [65]. The binary differential evolution (BDE) algorithm was introduced by Pampara et al. [66], and the trigonometric function is utilized to produce 0 − 1 string to map floating-point variables into binary numbers. For the feature selection issues, the primary vector is operated as a candidate feature subset and the feature subset is changed with the mutation and the crossover actions. The distance between interclass and intraclass samples is computed as the target function to rate the quality of the feature subset.

Suppose that the initial population *P*^0^=*X*^0^ for *i* = 1,…, *N* consists of *N* randomly selected individual solutions. In the mutation process, three vectors *X*_*r*1_,  *X*_*r*2_, and *X*_*r*3_ are randomly selected from each population for each vector *X*_*i*_, such that *r*1  ≠ *r*2  ≠ *r*3  ≠ *i*. *X*_*r*1_ is called a base vector. *X*_*r*2_ and *X*_*r*3_ individuals determine whether the *j*th bit of *X*_*r*3_ is flipped (*V*_*i*,*j*_ = 1 −  *X*_*i*,*j*_) or not. A crossover between the mutant *V*_*i*_ and its parent *X*_*i*_ determines the trial vector *U*_*i*_. Therefore, the difference vector is calculated as [65, 67]

(13) $$\begin{array}{c} \text{Difference }{\text{vector}}_{\text{id}}=\left\{\begin{array}{cc} 0, & \text{ if }X_{r1d}=X_{r2d},\\ X_{r1d}, & \text{otherwise.} \end{array}\right) \end{array}$$

The mutant vector is then computed as follows:

(14) $$\begin{array}{c} V_{\text{id}}=\left\{\begin{array}{cc} 1, & \text{ if difference }{\text{vector}}_{\text{id}}=1,\\ X_{r3d}, & \text{otherwise}, \end{array}\right) \end{array}$$

where *i* and *d* are the vector order and search space dimension, respectively. Moreover, the trial vector *U* is produced as follows:

(15) $$\begin{array}{c} U_{\text{id}}=\left\{\begin{array}{cc} V_{\text{id}}, & \text{ if }\left(\text{rand}\leq CR\right)\text{ or }d=\text{and,}\\ X_{\text{id}}, & \text{otherwise,} \end{array}\right) \end{array}$$

where *X* is the vector, rand is a random number in [1,  *D*], and CR is a constant crossover rate in [0, 1]. In the selection phase, if the fitness of the trial vector is better than the current vector, it will be substituted for the next generation. In the current study, the maximum number of iterations is fixed to 100, the number of vectors is set to ten, and CR = 0.9. Besides, the total number of features in the particle is set as many as all features in the dataset.

#### 2.5.3. Firefly Algorithm

The firefly algorithm (FA) is inspired by the flashing behavior of fireflies [68]. Fireflies attract the opposite-sex counterparts by exploiting this flashing behavior. However, in the mathematical model of the FA, the fireflies are unisex, and each firefly may attract other fireflies. The charm of a firefly is equal to its brightness, and, for both fireflies, the brighter one will attract the other. Therefore, the firefly with less brightness flies towards a brighter one. The brightness intensity is inversely proportional to the distance. The distance between any two fireflies (*i* and *j*) at *x*_*i*_ and *x*_*j*_ is calculated by the Cartesian distance as follows [68]:

(16) $$\begin{array}{c} r_{ij}=\left\|x_{j}-x_{i}\right\|=\sqrt{\overset{D}{\underset{k=1}{\sum }}{\left(x_{ik}-x_{jk}\right)}^{2}}, \end{array}$$

where *D* is the dimension. The attractiveness of a firefly decreases exponentially as the distance increases. In the FA, the primary form of attractiveness function *β*(*r*) is given by

(17) $$\begin{array}{c} \beta \left(r\right)=\beta_{0}e^{-\gamma r^{2}}. \end{array}$$

Here *r* and *β*(*r*) indicate the distance and the attractiveness at *r* between two fireflies, respectively. The original brightness (*β*_0_) is the attractiveness at *r* = 0 and *γ* is a fixed light absorption coefficient. The movement of a firefly  *i* is specified as follows:

(18) $$\begin{array}{c} X_{i}\;=X_{i}\;+\;\beta \left(r\right)\left(X_{\text{best}}\;–\;X_{i}\right)+\;\alpha \left(\frac{\text{rand}}{2}\right). \end{array}$$

The second term is owing to the attraction; *X*_best_ is the location of the most attractive firefly. Besides, the third term is randomization with *α* and rand  is *U*[0,  1]. When the firefly *i* moves towards firefly *j*, the position of firefly *i* is changed from a binary number to a floating-point number. Therefore, the sigmoid function maps the position in [0,  1].

(19) $$\begin{array}{c} S\left(x_{\text{ik}}\right)=\frac{1}{1+e^{-x_{\text{ik}}}}. \end{array}$$

Then the position of firefly *i* is updated as follows:

(20) $$\begin{array}{c} x_{\text{id}}=\left\{\begin{array}{cc} 1, & \text{if }\rho_{\text{id}}\leq S\left(x_{\text{id}}\right),\\ 0, & \text{otherwise,} \end{array}\right) \end{array}$$

where *x*_id_ represents each bit of the dimension vector *X*_*i*_ and *ρ*_id_ is *U*[0,1]. This guarantees that each bit will be either 0 or 1 [69]. In our study, the FA is iterated 100 times by using six fireflies and setting *α*= 0.5 and *γ*=0.

#### 2.5.4. Genetic Algorithm

The genetic algorithm (GA) is a heuristic search algorithm inspired by Darwin's theory of evolution [70]. GA starts with a set of solutions (chromosomes) called population. A new population is initiated by using these chromosomes. This is motivated by the hope that the new population will be superior to the former one. The chromosomes have been chosen based on their fitness to create new chromosomes (offspring). Crossover and mutation are the two leading operators of GA. There are different crossover approaches, such as roulette wheels, tournaments, and rank, which pick genes from parent chromosomes and create new offspring. After crossover, a mutation occurs to prevent falling into the local optimum. Mutations change the new offspring randomly. This is iterated until the population size or improvement of the best solution is met [71].  Figure 4 summarizes the GA steps.

GA has four basic parameters: the number of chromosomes (*N*), the maximum number of generations (*T*), the crossover rate (CR) probability, and the probability of mutation rate (MR). CR determines how many times the crossover needs to be done. If there is no crossover, the offspring is just a copy of the parents. If there is a crossover, some parts of the parent's chromosome form the offspring [70, 71]. Mutation probability indicates how many times the parts of the chromosome mutate. If there is no mutation, the offspring will be transplanted without any change. If a mutation is exploited, a part of the chromosome will be modified. We use mutations to prevent the GA from crashing in the extreme, but it does not need to happen very often because the GA turns into a random search. Here, we used GA to select the best features using ten chromosomes and 100 generations. Besides, CR and MR probabilities are initialized to 0.8 and 0.01, respectively, and the number of genes is the total number of features in the dataset.

#### 2.5.5. Grey Wolf Optimization

Grey wolf optimization (GWO) is a recent population-based optimization approach, which simulates the hunting process of grey wolves in nature [72]. Grey wolves more often prefer to live and hunt in a pack with an average of 5∼12 wolves and pursue stringent *t* rules in a hierarchy. The most influential wolf in decision-making is named alpha (*α*), which leads the whole pack. The betas (*β*), probably the best nominees for the alpha, are subordinates of alpha which support it in decision-making or other activities and reinforce its decisions among other lower-level wolves. The omega is the next level of the beta in a hierarchy. The omega (*ω*) wolves play the role of scapegoat. They must surrender to all dominant wolves. They are the last wolves permitted to feed. If a wolf in the pack does not belong to any group, it is called a delta (*δ*) wolf. Deltas need to submit alpha and beta, but they dominate the omega [67, 72].

In GWO, each wolf updates its position according to the distance from the updated prey position as the best three solutions of alpha, beta, and omega. The distance between each wolf and the prey $\overset{⟶}{\left(D\right)}$ is defined as

(21) $$\begin{array}{c} \overset{⟶}{D}=\left|\overset{⟶}{C}.\;{\overset{⟶}{X}}_{P}\left(t\right)-\overset{⟶}{X}\left(t\right)\right|,\\ \overset{⟶}{C}=2.\;\overset{⟶}{r_{2}}\text{ ,} \end{array}$$

where $\overset{⟶}{C}$ is the coefficient vector and ${\overset{⟶}{X}}_{P}\left(t\right)$ and $\overset{⟶}{X}\left(t\right)$ indicate the position vectors of the prey and a wolf, respectively. Also, *t* shows the current iteration and $\overset{⟶}{r_{2}}$ is a random vector in the [0, 1] interval.

(22) $$\begin{array}{c} \overset{⟶}{D}=\left|\overset{⟶}{C}.\;{\overset{⟶}{X}}_{P}\left(t\right)-\overset{⟶}{X}\left(t\right)\right|,\\ \overset{⟶}{C}=2.\;\overset{⟶}{r_{2}}\text{ .} \end{array}$$

A prey's location is determined by

(23) $$\begin{array}{c} \overset{⟶}{X}\left(t+1\right)={\overset{⟶}{X}}_{P}\left(t\right)-\overset{⟶}{A}\;.\overset{⟶}{D},\\ \overset{⟶}{A}=2\overset{⟶}{a}.\overset{⟶}{r_{1}}-\overset{⟶}{a}, \end{array}$$

where $\overset{⟶}{A}$ is a coefficient vector, $\overset{⟶}{r_{2}}$ is a random vector in the interval [0, 1], and the members of $\overset{⟶}{a}$ are linearly decreased from 2 to 0 during the optimization phase. In addition, the position of wolves is updated as follows:

(24) $$\begin{array}{c} \overset{⟶}{D_{\alpha }}=\left|\overset{⟶}{C_{1}}\cdot \overset{⟶}{X_{\alpha }}-\overset{⟶}{X}\right|,\\ \overset{⟶}{D_{\beta }}=\left|\overset{⟶}{C_{2}}\overset{⟶}{X_{\beta }}-\overset{⟶}{X}\right|,\\ \overset{⟶}{D_{\delta }}=\left|\overset{⟶}{C_{3}}\overset{⟶}{X_{\delta }}-\overset{⟶}{X}\right|,\\ \overset{⟶}{X_{1}}=\overset{⟶}{X_{\alpha }}-\overset{⟶}{A_{1}}.\overset{⟶}{\left(D_{\alpha }\right)},\\ \overset{⟶}{X_{2}}=\overset{⟶}{X_{\beta }}-\overset{⟶}{A_{2}}.\overset{⟶}{\left(D_{\beta }\right)}\text{, }\\ \overset{⟶}{X_{3}}=\overset{⟶}{X_{\delta }}-\overset{⟶}{A_{3}}.\overset{⟶}{\left(D_{\delta }\right)},\\ \overset{⟶}{X}\left(t+1\right)=\frac{\overset{⟶}{X_{1}}+\overset{⟶}{X_{2}}+\overset{⟶}{X_{3}}}{3}. \end{array}$$

Wolves update their positions to the actual values in the potential search space limited explicitly by the problem constraints. Nevertheless, for some issues, variables and search space are restricted explicitly to binary values [0, 1]. Feature selection is a binary issue and a feature subset is shown as a binary vector and each member in the vector specifies a single feature. A value of 1 for each feature represents that it is selected, and vice versa. Therefore, in binary GWO, variables and search space are mapped from real values to binary values using the sigmoid function [72].

(25) $$\begin{array}{c} v_{\text{sol}}^{d}\left(t\right)=A_{1}^{d}.D_{\text{sol}}^{d},\\ T\left(v_{\text{sol}}^{d}\left(t\right)\right)=\frac{1}{1+e^{-10\;vd/\text{sol}\left(t\right)}-0.5}. \end{array}$$

Therefore, for a solution *x* and dimension *d*, we have [72]

(26) $$\begin{array}{c} x_{d}^{\text{new}}=\left\{\begin{array}{cc} 1, & x_{d}^{\text{old}}+T\left(v_{sol}^{d}\left(t\right)\right)\geq 1,\\ 0, & \text{ otherwise.} \end{array}\right) \end{array}$$

In our study, the binary GWO algorithm is iterated 100 times by using ten wolves.

#### 2.5.6. Particle Swarm Optimization

Binary particle swarm optimization (PSO) [73] is the discrete version of the PSO algorithm [74] which solves optimization problems based on the social behavior of animals such as the mass movement of birds and fish. Every single solution in the PSO is assumed as a particle. Every particle tries to find the best position over time. It adapts its position with regard to its own experience and the experiences of its neighbors consisting of the current velocity and position and the best prior position experienced by it and its neighbors. This process is performed repeatedly until a predetermined minimum error is reached or up to a certain number of repetitions and so on [67]. The last position of ant particle *i*  that previously had good fitness is stored as the best person (*p*_besti_), and the best particle position that has the best fitness among the population is stored as the best global (*g*_besti_), where *r*_1_ and *r*_2_ are random values in the range of (0, 1) and *c*_1_ and *c*_2_ are cognitive and social parameters, respectively.

In binary PSO, particle positions are modeled into the bit string to limit the velocity in the range [0,1]. Furthermore, the velocity of a particle is defined as the probability that a particle might change its state to one. Traditional binary PSO and most of its variants use different probability functions to cope with discrete optimization problems. The input parameters of binary PSO are the number of iterations (*T*), the number of particles (*N*), cognitive learning factor (*c*_1_), the social learning factor (*c*_2_), the maximum bound on inertia weight (*ω*_Max_), the minimum bound on inertia weight (*ω*_Min_), the maximum velocity (*V*_Max_), and the total features in a particle. Also, *ω* is called the inertial weight and it plays the tuning role in global and local searches. In case that *d* is the dimension, the position and velocity vectors of the *i*th particle are deﬁned as *X*_*i*_=(*x*_1_,  *x*_2_,…,  *x*_id_) and *V*_*i*_=(*v*_1_,  *v*_2_,…, *v*_id_).

The equation to update the velocity of each particle is as follows:

(27) $$\begin{array}{c} v_{\text{id}}^{\text{new}}=v_{\text{id}}^{\text{old}}+c_{1}r_{1}\left(p_{\text{best id}}-x_{\text{id}}^{\text{old}}\right)+c_{2}r_{2}\left(g_{\text{best id}}-x_{\text{id}}^{\text{old}}\right). \end{array}$$

By using the sigmoid function, the position will be updated according to the following equations:

(28) $$\begin{array}{c} S\left(v_{\text{id}}\right)=\frac{1}{1+e^{-v_{\text{id}}}}, \end{array}$$

(29) $$\begin{array}{c} x_{\text{id}}^{\text{new}}=\left\{\begin{array}{cc} 1, & \text{if }\rho_{id}\leq S\left(v_{\text{id}}^{\text{new}}\right),\\ 0, & \text{otherwise,} \end{array}\right) \end{array}$$

where *ρ*_id_  is *U*[0,1].

In the current study, the maximum iterations are kept to 100, the total particle in population is set to ten, and the total number of features in the particle is set as many as all features in the dataset. Cognitive and social factors (*c*_1_ and *c*_2_) are assigned the value of 2. Also, *ω*_Min_, *ω*_Max_, and *V*_Max_ are initialized by 0.4, 0.9, and 6, respectively.

### 2.6. Classification

After selecting the significant features, these are fed to the classifiers for evaluating the performance of the proposed framework. In the present study, the results of classifiers are reported by deploying a tenfold cross-validation strategy 2541654, which is used to divide the dataset into ten equal subsets. After that, at any time, one subset will be used as test data and the remaining nine subsets will be used as training data for the classifiers. In other words, any EEG signal of the dataset is used nine times as training data and once as test data.

The label of test data is clear, so there are four conditions for any test data after the classification [39–41, 75]:

  True positive (TP): if a test signal with a focal label is correctly classified in the focal group
  True negative (TN): if a test signal with a nonfocal label is correctly classified in the nonfocal group
  False positive (FP): if a test signal with a nonfocal label is incorrectly classified in the focal group
  False negative (FN): if a test signal with a focal label is incorrectly classified in the nonfocal group

The following equations are used to evaluate the classifier ACC, sensitivity (SEN), and specificity (SPE) [4, 23, 75]:

(30) $$\begin{array}{c} \text{ACC}=\frac{T_{\text{TP}}+T_{\text{TN}}}{T_{\text{TP}}+T_{\text{TN}}+T_{\text{FP}}+T_{\text{FN}}}\times 100,\\ \text{SEN}=\frac{T_{\text{TP}}}{T_{\text{TP}}+T_{\text{FN}}}\times 100,\\ \text{SPE}=\frac{T_{\text{TN}}}{T_{\text{TN}}+T_{\text{FP}}}\times 100, \end{array}$$

where *T*_TP_, *T*_TN_, *T*_FP_, and *T*_FN_ are the total numbers of TP, TN, FP, and FN after ten times training and testing classifier. ACC shows the ability of the classifier to discriminate F and NF signals. Also, SEN shows the ability of classifiers in the detection of focal EEG signals. On other hand, SPE shows the ability of classifiers in the detection of nonfocal EEG signals.

In this work, six classifiers, namely, KNN, SVM, FFNN, CFNN, GRNN, and RNN, are used for classifying the EEG signals in focal and nonfocal groups. In the following subsections, we describe these used classifiers.

#### 2.6.1. *K*-Nearest Neighbor (KNN)

The well-known *K*-nearest neighbors (KNN) algorithm is a supervised classifier with very easy implementation [6, 13, 23]. In the KNN algorithm, every test data is classified with *K*-closed neighbors. That way, test data belongs to the group which has more members in *K*-closed neighbor. The number of *K* and distance computation methods are the two main parameters of the KNN classifier. In this work, city-block distance with various numbers of *K* ranging from 1 to 9 with a step equal to 1 was used to attain the best results.

#### 2.6.2. Support Vector Machine (SVM)

Nowadays, the support vector machine (SVM) algorithm is becoming one of the most widely used classifiers in biomedical machine learning applications. The SVM algorithm maps the features in a high dimensional space by kernel function and constructs an optimum hyperplane for separating the classes [6, 12, 14, 22]. In the new higher-dimension space, features in each class are near together and are far away from the other class. In this work, the radial basis function (RBF) is used as kernel [13] and the sigma values of RBF vary from 0.1 to 1.5 by the step size of 0.1 to attain the best results.

#### 2.6.3. Feed-Forward Neural Network (FFNN)

In feed-forward neural networks (FFNN), neurons are arranged in multiple layers and signals are forwarded from input to output. When an error occurs, these neurons are returned to the previous layer and weights are adjusted again to reduce the error chances. In this study, we use the tan-sigmoid transfer function, a single hidden layer with ten empirically chosen neurons, and the Levenberg-Marquardt algorithm for fast training [37, 39–41].

#### 2.6.4. Cascade-Forward Neural Network (CFNN)

In cascade-forward neural networks (CFNN), neurons are interlinked with previous and subsequent layers of neurons [76]. For example, a three-layer CFNN represents the direct connections between layer one and layer two, between layer two and layer three, and between layer one and layer three; that is, neurons are directly and indirectly connected in the input and output layers. These additional connections help to achieve a better learning speed for the required relationship. Like FFNN, in CFNN, we have utilized the tan-sigmoid transfer function, one hidden layer with ten neurons selected by a hit and trial manner, and Levenberg-Marquardt method for quick learning.

#### 2.6.5. Generalized Regression Neural Network (GRNN)

The general regression neural network (GRNN) is a single-pass neural network that uses a Gaussian activation function in the hidden layer. GRNN consists of input, hidden, summation, and division layers. The classification accuracy of GRNN is largely dependent on the accurate value of the spread factor. In this study, the spread factor is fixed to 1 after several experiments for the classification of focal and nonfocal EEG signals [1, 77, 78].

#### 2.6.6. Recurrent Neural Network (RNN)

In recurrent neural networks (RNN), neurons can flow in a circle because this network has one or more feedback links. The characteristics of RNN allow the system to process temporarily and recognize the trends. In this study, we are implementing Elman recurrent neural network, which is the prevalent form of RNN. For quick training of the model, the Levenberg-Marquardt method and single hidden layer with ten empirically selected neurons are utilized [77].

## 3. Results

### 3.1. Preprocessing

Each signal of the Bern-Barcelona dataset has two different time series which are “*X*” and “*Y*.” For noise reduction, “*X*-*Y*” is recommended as an input signal in the previous studies [6, 11, 17, 34]. For this reason, we have also used the “*X*-*Y*” time series as an input signal. In [23, 32], the effect of differential operators in focal and nonfocal EEG signal detection has been discussed and suggested to use different features. For that, we have applied the differential operator to the “*X*-*Y*” time series before the TQWT decomposition.

### 3.2. Selection of TQWT Parameters

The accuracy of a classifier and involved intense calculations are directly dependent on the selection of optimal values of *Q*, *r*, and *J* of TQWT transform. In other words, the selection of the optimal value of these parameters is an important step before signal decomposition. We used three steps for setting the parameters of TQWT. In the first step, *Q*, *r*, and *J* are assumed to be fixed for choosing the best classifier. In the second step, *J* is assumed to be fixed for setting the optimum values of *Q* and *r* parameters. In the third step, by having the optimum values of *Q* and *r*, the optimum value of *J* is found.

*First Step*. For choosing the optimal values of TQWT parameters, the values of *Q* and *r* were set to 2 and the value of *J* was selected to be 5. Then entropy-based features were extracted from subbands and fed to KNN, SVM, FFNN, CFNN, RNN, and GRNN classifiers. The ten-fold cross-validation strategy has been employed during the training and testing of the classifiers.  Figure 5 shows the resulting classification ACC by these features for various classifiers.

*Second Step*. In this step, *Q* is varied from 2 to 10, *r* is varied from 2 to 5, and the value of *J* is kept fixed, which is 5. Then, the entropy-based features are extracted from subbands and fed to the CFNN classifier.  Figure 6 illustrates the resulting ACC for various numbers of *Q* and *r*.

It is evident from Figure 4 that the deployment of TQWT along with the CFNN classifier resulted in the highest classification ACC when the values of both *Q* and *r* were 3.

*Third Step*. By fixing *Q* and *r* to 3, the maximum decomposition level of TQWT is 35; so, we checked the resulting classification ACC for *J* from 5 to 35 and illustrated the results in Figure 7.

Figure 7 depicts that the ACC of the CFNN classifier is improved by increasing the decomposition level and maximum ACC is achieved when the value of *J* is 26. Finally, the optimum values of *Q*, *r*, and *J* are found to be 3, 3, and 26, respectively, which lead up to the best classification performance. It should be noted that, by selecting *J* to be 26, input EEG signals are decomposed to 27 subbands, 1 approximation and 26 details, in such a way that subband1 to subband26 are detail1 to detail26 and subband27 is approximation 26.

Furthermore, by using the selected optimum values for *Q*, *r*, and *J* parameters, Figure 8 shows the designed TQWT filter bank in the frequency domain and Figure 9 shows the decomposed TQWT subbands.

### 3.3. Feature Extraction

The mean and standard deviation of extracted entropy-based features for focal and nonfocal EEG signals are written in Table 1. It is clear that the values of entropy-based features for the focal group in all subbands except for details 1, 2, and 3 are lesser than those of the nonfocal group. Also, the standard deviation of extracting entropy-based features in the focal group was less than that of the nonfocal group. Since the entropy is a parameter for the quantification of chaotic behavior of signal, we can say that lower mean and standard deviation value of entropies in the focal group indicates less random (more rhythmic) behaviors of the focal EEG signals in comparison to nonfocal EEG signals.

### 3.4. Feature Selection and Classification

The statistically significant features for focal signal detection have been obtained using a *p* value in previous studies [6, 11, 13–17, 19, 22, 23, 32–34]. In mentioned studies, the features with a *p* value of less than 0.05 were selected as significant features. Generally, a lesser *p* value indicates a better ability to extract features in binary classification. We deployed the KWS test to compute the *p* value of extracted entropy-based features from TQWT subbands, and the “Kruskal-Wallis” MATLAB function is used for computation purposes.

It is obvious from Table 1 that all of the extracted entropy-based features show good discrimination between focal and nonfocal signals and the *p* value for all features is less than 0.05. In other words, we can use all of the entropy-based features in the classification of focal and nonfocal EEG signals. So, these features were fed to KNN, SVM, FFNN, CFNN, RNN, GRNN, and RNN classifiers. The resulting ACC, SEN, and SPE and the comparison of classifier performances for all of the extracted entropy-based features are given in Table 2. Though by using the entropy-based features a good average classification ACC of 94.77% has been achieved by exploiting CFNN classifier, the feature vector has 108 arrays (i.e., four entropy features extracted from 27 subbands) which lead the proposed method to be more complex. For this reason, we tested various optimization algorithms as a feature selection method for decreasing the arrays of the input feature vector to reduce the complexity of the proposed method.

The resulting classification ACC, SEN, and SPE for classifiers with the feature selected by the BBA algorithm are written in Table 3. It is clear from Table 3 that the classifier performance for selected features of the BBA algorithm has increased in comparison to when all entropy-based features are fed to classifiers, although the feature vector has less arrays. So, the BBA algorithm cannot improve the performance of the proposed method. It should be noted that the feature vector in FFNN classifier which resulted in 90.62% classification ACC has 34 arrays. In other words, the BBA algorithm discards 74 features (i.e., BBA algorithm made the feature vector 79.92% smaller). The feature vector arrays selected by the BBA algorithm and fed to FFNN classifier were the LE entropy of details 7, 9, 11, 12, 14, 16, and 18, the LL2 entropy of details 5, 7, 11, 17, 18, 19, 20, and 23, approximation 26, the SURE entropy of details 6, 7, 9, 14, 15, 16, 19, 20, 22, and 26, and the TH entropy of 3, 4, 13, 14, 15, 16, 24, and 26.

In the same way, the selected entropy-based features by the BDE algorithm are fed to classifiers. The performance of the classifiers with these selected features is given in Table 4. The resulting classification ACC, SEN, and SPE for selected features by the BDE algorithm are slightly different from the resulting classification ACC, SEN, and SPE for all entropy-based features. On the other hand, 93.81% ACC resulted in the CFNN classifier by 93 selected features, which indicated that BDE cannot significantly reduce the complexity of the proposed method. In other words, the BDE algorithm with CFNN fitness function just discards 15 features (i.e., BDE algorithm made the feature vector 16.2% smaller). The BDE algorithm with CFNN fitness function used from all entropy-based features for classification, except LE entropy of details 1, 2, 3, 5, 7, 8, 12, and 16, the LL2 entropy of detail 2, the SURE entropy of details 22 and 24, the TH entropy of details 4, 19, and 22, and approximation 26.

Furthermore, the performances of classifiers for selected features by the FA algorithm are given in Table 5. It can be understood that the results of classifiers with selected features by the FA algorithm are not very different from those in classification ACC, SEN, and SPE for all entropy-based features. In Table 5, the FFNN classifier resulted in 93.02% classification ACC, which is slightly higher than those of the other classifiers. On the other hand, the FA algorithm selected 52 features with the FFNN fitness function. The FA discards 56 features (i.e., FA algorithm made the feature vector 60.48% smaller) which leads the proposed method to be simpler. The selected features by FA algorithm with FFNN fitness function which made input feature vector arrays were LE entropy of details 6, 9, 11, 14, 15, 17, 18, 19, 22, 23, and 24 and approximation 27, LL2 entropy of details 4, 6, 8, 9, 10, 11, 12, 16, 17, 24, and 26 and approximation 27, SURE entropy of details 1, 2, 3, 4, 7, 8, 9, 11, 17, 22, 24, and 25 and approximation 27, and TH entropy of details 1, 2, 3, 4, 5, 6, 8, 9, 11, 15, 18, 20, 22, and 24 and approximation 26.

The performance of classifiers with selected features by GA is summarized in Table 6. The highest classification ACC for selected entropy-based features by using GA and CFNN classifier is 93.53%. GA with CFNN fitness function selected 57 features, which means the GA discards 51 features (i.e., GA made the feature vector 55.08% smaller). The selected features by GA with CFNN fitness function were LE entropy of details 6, 9, 10, 12, 14, 15, 16, 17, 18, 19, 21, 22, 23, 24, 25, and 26 and approximation 27, LL2 entropy of details 1, 2, 4, 8, 9, 10, 11, 17, 18, 19, 20, 23, and 25, SURE entropy of details 1, 2, 3, 4, 5, 8, 10, 11, 15, 18, 19, and 20, and TH entropy of details 1, 2, 4, 7, 9, 10, 12, 13, 16, 17, 21, 23, 25, and 26 and approximation 26, which made the input feature vector arrays.

The classifier's performance for selected entropy-based features by the GWO algorithm is given in Table 7. It is clear from Table 7 that the selected entropy-based features by the GWO algorithm with the CFNN classifier resulted in 93.45% classification ACC which is higher than those of other classifiers. The GWO algorithm with the CFNN fitness function selected 88 entropy-based features. In other words, the feature vector has 88 arrays and the GWO algorithm discards 20 features (i.e., GWO algorithm made the feature vector 21.60% smaller). The discarded features by GWO algorithm with CFNN were LE entropy of details 1, 2, 3, 5, 7, and 8, LL2 entropy of details 7, 11, 12, 18, 22, and 26 and approximation 26, SURE entropy of details 12 and 22, and TH entropy of details 15, 20, 22, 25, and 26.

The resulting classification ACC, SEN, and SPE for selected features by the PSO algorithm are shown in Table 8. It is evident from Table 8 that selected entropy-based features by the PSO algorithm improved the performance of the classifier. The best performance resulted from the CFNN classifier, which achieved a perfect average classification ACC of 97.68% for 63 entropy-based features selected by the PSO algorithm with CFNN fitness function. The selected entropy-based features by PSO algorithm with CFNN fitness function were LE entropy of details 4, 7, 9, 10, 11, 14, 15, 16, 17, 18, 19, 20, 21, 22, 23, and 24 and approximation 26, LL2 entropy of details 3, 5, 6, 8, 9, 10, 11, 12, 15, 16, 20, 21, 22, 25, and 26 and approximation 26, SURE entropy of details 1, 2, 4, 7, 8, 9, 10, 12, 14, 18, 19, 20, 22, 24, and 26, and TH entropy of details 1, 5, 6, 9, 11, 13, 14, 15, 16, 17, 18, 21, 22, 23, and 24. The PSO algorithm discarded 45 features (i.e., PSO algorithm made the feature vector 48.60% smaller). A comparison between the performances of classifiers and feature selection methods is illustrated in Figure 10.

From Tables 2–8 and Figure 11, we can say that PSO is a significant feature selection method and FFNN, CFNN, and RNN classifiers are more appropriate than the other feature selection methods and classifiers for focal EEG signal detection application, respectively. We should note that although the KWS test resulted in acceptable classification performance in comparison to most of the feature selection methods, it did not increase the feature vector arrays and used all extracted entropy-based features.

The receiver operating characteristic (ROC) value for the classifiers for each feature section algorithm is shown in Figure 11. It is clear from Figure 11 that the area under the curve of the PSO algorithm is significantly higher than those of the other feature selection algorithms. The computational time of the algorithm for all signals of the Bern-Barcelona EEG dataset including preprocessing and differencing, the generation of TQWT filter bank, subband separation, and extraction of LE, LL2, SURE, and TH entropies as features using i5-M480 CPU (2.67 GHz), 6 GB RAM, and MATLAB 2014a is 215.6 seconds (i.e., 0.0287 seconds for any input signal) which indicates the robustness of the proposed method. The Bern-Barcelona dataset has more than 41.6 hours of EEG signals and the CFNN classifier required only 0.17 s for the classification of an input test signal. The algorithm time can be further reduced by using a powerful machine and another computationally efficient software package.

## 4. Discussion

The correct classification of focal and nonfocal EEG signals is directly linked to minimizing the surgical complications for the patients who are immune to antiepileptic drugs. In the present study, we proposed a computer-based method for the correct classification of focal and nonfocal EEG signals. The Bern-Barcelona dataset was used for the evaluation of the proposed method. Each file of the Bern-Barcelona dataset has two signals, namely, “*X*” and “*Y*,” recorded from adjacent channels. In the proposed framework, the “*X-Y*” signal is applied on differencing operator and decomposed using TQWT in optimal condition by setting *Q*, *r*, and *J* to 3, 3, and 26, respectively. LE, LL2, SURE, ad TH entropies are extracted from TQWT subbands as features. The performance of several feature selection and classification methods is checked among which PSO algorithm and CFNN classifier are chosen as the feature selection and classification methods. A proposed framework achieved an average classification ACC of 97.68%, SEN of 97.26%, and SPE of 98.11% in a ten-fold cross-validation strategy. Boxplots of selected features by PSO algorithm with CFNN fitness function are shown in Figure 12.

We found that proposed entropy-based features are significantly good parameters in the classification of focal and nonfocal EEG signals since their corresponding *p* value was less than 0.05 for all subbands as depicted in Table 1. Furthermore, the lower mean and standard deviation values of entropies in the focal group indicate less randomness of the focal EEG signals in comparison to nonfocal EEG signals as reported in previous studies [6, 10, 11, 22, 23, 25, 33, 34]. We showed that the performance of heuristic algorithms in the reduction of feature vector arrays is better than the KWS test, although features selected by some heuristic algorithms resulted in lesser classification ACC.

We compared the performance of the proposed method with those of the state-of-the-art methods which used the same dataset as ours and details are demonstrated in Table 9. In [10], delay permutation entropy with different delay lags has been extracted as discrimination features from EEG signals and applied to the SVM classifier which resulted in classification ACC of 84% and 75% for 50 and 750 EEG signals, respectively. They found that the value of delay permutation entropy for focal EEG signals is significantly more than that of the nonfocal EEG signals. In [15], sample entropy and variance of instantaneous frequencies of intrinsic mode functions (IMFs) have been computed as a feature and fed to the least-square SVM (LS-SVM). The authors therein obtained 85% classification ACC for 50 EEG signals.

In [16], average Shannon entropy, average Renyi's entropy, average approximate entropy, average sample entropy, and average phase entropy of IMFs were computed as features which resulted in 87% classification ACC for 50 EEG signals. They computed the *p* value for extracting features and found that the entropies for IMFs can be used as a useful parameter for focal EEG signal detection. In similar research [17], nonlinearity of EEG signals has been measured by centered correntropy, information potential, and LE and SURE entropies of the IMFs as a feature and applied to SVM classifier which resulted in 89% classification ACC for 50 EEG signals. Also, the calculations of their method were very intense. In [18], the spectrum of EEG signals was obtained by S-transform and then the time-frequency entropy of spectrum was used as a feature which resulted in 86% classification ACC for 50 EEG signals. Although the reported classification ACC was not significantly higher, it resulted in only one feature being used. Besides that, the authors therein found that a spectrogram of EEG signals can be used as significant parameters for focal EEG signal detection. In [19], Daubechies wavelet of order 4 decomposed the EEG signals to four levels, and entropy-based features have been extracted from DWT coefficients of EEG signals for detecting focal EEG signals which resulted in 84% classification ACC for 50 EEG signals. Although the reported classification ACC of their method was not significantly higher and the calculations for extracting features were heavy, on the other hand, the authors therein proposed a novel integrated discrimination index for focal and nonfocal EEG signal classification based on these features. In [20], EEG signals have been decomposed to coefficients and nine linear features extracted from coefficients and fed to SVM classifier which achieved 83.7% classification ACC for 3750 EEG signals. The authors therein tested the performance of extracting features for fifty-four mother wavelets from seven families, namely, Haar, Daubechies, Meyer, Coiflets, Biorthogonal, Reverse biorthogonal, and Symlets, and found that the performance of classifiers is not dependent on the choice of wavelet family, and it is more dependent on decomposition levels.

In [6], EMD was used for extraction of the first two IMFs of EEG signals; then DWT decomposed IMFs into four levels. In other words, EEG signals have been decomposed by EMD-DWT to ten subbands (i.e., one approximation and four details for IMF1 and IMF2). Then Shannon and Renyi and LE entropies of subbands were calculated as features and fed to KNN classifier which obtained classification ACC of 90.5% and 89.40% for 50 and 3750 EEG signals, respectively. They reported these results by considering 20% of EEG signals as training data and the other 80% as testing data in the classification process. They found that first IMFs (i.e., highest frequencies of EEG signals) and LE entropy are more significant in the detection of focal and nonfocal EEG signal classification. In [31], the same authors expanded the features in the VMD-DWT domain and reported 95.2% classification ACC using the SVM classifier for 3750 EEG signals. In [14, 22–24], EEG signals are separated into rhythms by Fourier transform [14] and empirical wavelet transform [22–24]. In [14], the mean frequency and root mean square of EEG signals were derived as a feature and fed to LS-SVM classifier which obtained 89.7% and 89.5% classification ACC for 50 and 750 EEG signals, respectively. The authors therein found that frequency-based features extracted from rhythms are usable in focal detection.

In [24], the nonlinearity of EEG signals rhythms in EWT domain was computed as feature and fed to classifier in which classification ACC of 93% and 82.6% were reported for 50 and 3750 EEG signals, respectively. In [27], a method based on the combination of the EEG rhythms in FBSE-EWT domain and sparse autoencoder-support vector machine is proposed for detection of focal EEG signals which resulted in perfect classification ACC of 100%. In another method based on deep learning [21], the time-frequency matric of EEG signal was computed in Fourier synchrosqueezing transform domain (FSST) and wavelet synchrosqueezing transform domain (WSST) and fed to a deep convolutional neural network (CNN) for the classification. This method could achieve classification ACC of 99%. Recently, a method based on Taylor-Fourier filter bank implemented with O-Splines has been proposed to extract the EEG rhythms [5]. In [29], a method based on decomposition of the EEG signal by sliding mode-singular spectrum analysis (SM-SSA) with sparse autoencoder hidden layer and radial basis function neural network (SAE-RBFN) classifier was proposed, which resulted in maximum classification ACC of 99.11%. In [28], mixture correntropy and exponential energy of subbands in FBSE-fTF-cwt domain were extracted as features and fed to a LS-SVM classifier; the authors therein reported average classification ACC of 95.85%.

In [22, 23], two-dimensional (2D) rhythms were drawn using phase space reconstruction [22] and second-order difference plot [23], respectively, in which the 2D illustration of EEG signals of the focal group in both methods had a more regular shape as compared to the nonfocal group which can be due to synchronous response from the neighboring neurons of the epileptogenic area which gives rise to focal EEG signals. This concept is reported in most of the previous research with other methods [6, 10, 11, 22, 23, 25, 33, 34] as well. In the present study, the mean and standard deviation of entropies for focal groups are less than those for nonfocal group, which indicate that the behaviors of focal EEG signals are less random and more rhythmic in comparison to the nonfocal EEG signals as described in Section 3.4.

In [33], the multiscale entropy of TQWT coefficients was extracted as features from EEG signals and fed to LS-SVM classifier which resulted in 84.67% classification ACC for 3750 EEG signals. Furthermore, in [34], *K*-nearest neighbor entropy estimator, centered correntropy, and fuzzy entropy of TQWT coefficients were extracted as features from EEG signals and fed to LS-SVM classifier, which achieved 95% classification ACC. In [33, 34], TQWT decomposed the focal and nonfocal EEG signals to 16 levels (i.e., *J* = 16), which resulted in 17 subbands. In our study, EEG signals are decomposed to 26 levels, which resulted in 27 subbands, which are more than those in the works in [25, 26], but, in our study, the time required for feature extraction from all subbands is significantly less as compared to those in the works in [25, 26] because they used multiscale entropy [33], *K*-nearest neighbor entropy estimator, centered correntropy [3, 24], and fuzzy entropy [34] which involve heavy calculations, while we deployed LE, LL2, SURE, and TH entropies that have very simple calculations leading our system to be time-efficient.

It is clear that the proposed method could achieve better classification ACC in comparison to most of the studies [6, 10–20, 22–26, 28, 30–34] in literature, but its classification ACC is less [21, 27, 29]. The proposed method in [21] needs to use two time-frequency analyses and deep learning technique whereby the value of calculation will be higher than that of our method. On the other hand, the proposed frameworks in [27, 29] could achieve better classification ACC with either lesser calculation [29] or fewer features, which shows the superiority of these methods compared with the proposed framework.

The advantages of the proposed framework over previous studies are enlisted as follows:

1. This is the first study to compare the performances of several feature selection algorithms and classifiers for focal and nonfocal EEG signal classification.
2. We have evaluated the performance of the proposed framework by using the entire Bern-Barcelona dataset (i.e., 3750 focal and 3750 nonfocal) while in [13, 15–19, 23] just 100 EEG signals (i.e., 50 focal and 50 nonfocal) have been used for evaluation of their methods.
3. We only used four entropies for classification of focal and nonfocal EEG signals, but in [16] six, in [19] seven, in [20] nine, in [11] fifty-two, and in [12] twenty-one various types of features have been computed for classification, which makes their studies computationally expensive.
4. Our results are reported in a ten-fold cross-validation strategy for ensuring the reliable classification performance of classifiers.
5. The proposed framework requires less than 0.2s for classifying any input EEG signals in focal or nonfocal groups which made our method time-efficient.
6. In [19], results have been reported with 10% standard deviation, while in our study, the results have around 3% standard deviation which indicates the robustness of our proposed method.
7. The proposed method can be deployed widely before surgery in hospitals as it is cost-effective and easily implementable with a computer and an EEG acquisition system.
8. The proposed method can detect focal EEG signals accurately without human intervention and errors.

Although the proposed method has the above-mentioned merits over the already existing methods, the main limitation of the present study is that the used Bern-Barcelona dataset has only EEG signals of five patients. In the future, the study would be extended by using the datasets involving a bigger number of patients.

## 5. Conclusion

The physicians can localize the brain surface before surgery by visual inspection of EEG signals. The correct classification of focal and nonfocal EEG signals by physicians for a long time is very hectic and time-consuming and may be prone to human errors. Thus, a computer-based system for distinguishing focal and nonfocal EEG signals with significant ACC is desirable. In the present study, we proposed a method based on entropy-based features extracted from TQWT subbands. Several feature selection, machine learning, and neural network classifiers were evaluated for discrimination of focal and nonfocal EEG signals evaluated on the Bern-Barcelona dataset with more than 41.6 hours of EEG data. The proposed TQWT-based method with different entropy-based features selected with the PSO method and classified by the CFNN resulted in classification ACC of 97.68%, which is higher than those of the previous methods. In the future, the performance of the proposed method is recommended for other biomedical signals to detect abnormal behaviors.

## Figures and Tables

**Figure 1:** Comparison of the normal brain with partial (focal) seizure and generalized seizure brains and their EEG signals.

**Figure 2:** The block diagram of the proposed method.

**Figure 3:** The first and second rows from left to right show the “*X*,” “*Y*,” “*X*-*Y*,” and differential for focal and nonfocal EEG signals, respectively.

**Figure 4:** Illustration of GA steps.

**Figure 5:** Resulting ACC for classifiers by fixing *Q* = *r* = 2 and *J* = 5. The highest classification ACC resulted from the CFNN classifier, so the CFNN classifier was chosen for setting the optimal value of TQWT parameters.

**Figure 6:** ACC of CFNN classifier for *J* = 5 and *Q* = 2, 3,…, 10 and *r* = 2, 3, 4, 5.

**Figure 7:** ACC of CFNN classifier for *Q* = *r* = 3 and *J* = 5, 6,…, 35.

**Figure 8:** TQWT filter bank in the frequency domain.

**Figure 9:** 27 decomposed subbands for focal and nonfocal EEG signals.

**Figure 10:** Illustration of each classifier performance for various feature selection methods.

**Figure 11:** ROC of classifiers for various feature selection techniques.

**Figure 12:** Boxplots of selected LE (a), LL2 (b), TH (c), and SURE (d) entropies in TQWT domain by PSO with CFNN fitness function.

**Table 1:** The mean ± standard deviation and *p* value for focal and nonfocal EEG signals. SB, D, and A are subband, detail, and approximation, respectively.

SB	LE entropy			LL2 entropy			SURE entropy			TH entropy		
	Focal	Non-focal	*p* value	Focal	Nonfocal	*p* value	Focal	Nonfocal	*p* value	Focal	Nonfocal	*p* value
D_1_	−3468 ± 1308	−2497 ± 2423	1.18*E* − 27	4.61 ± 1.05	4.76 ± 1.56	2.44*E* − 13	−3468 ± 1308	−2497 ± 2423	6.36*E* − 25	792 ± 639	1271 ± 1187	3.96*E* − 25
D_2_	971 ± 1322	1238 ± 2030	1.89*E* − 59	6.83 ± 1.07	7.01 ± 1.40	6.60*E* − 27	971 ± 1322	1238 ± 2030	6.33*E* − 66	2557 ± 651	2689 ± 1000	6.49*E* − 66
D_3_	2121 ± 765	2145 ± 1287	1.47*E* − 58	8.08 ± 1.18	8.24 ± 1.55	9.29*E* − 27	2121 ± 765	2145 ± 1287	3.85*E* − 65	2777 ± 377	2789 ± 634	3.88*E* − 65
D_4_	2149 ± 524	2098 ± 965	3.88*E* − 63	8.86 ± 1.28	8.72 ± 1.75	5.06*E* − 27	2149 ± 524	2098 ± 965	5.87*E* − 68	2502 ± 258	2477 ± 476	5.77*E* − 68
D_5_	1938 ± 398	1863 ± 774	9.61*E* − 59	9.19 ± 1.43	9.16 ± 1.88	1.53*E* − 15	1938 ± 398	1863 ± 774	3.72*E* − 68	2158 ± 197	2121 ± 381	3.76*E* − 68
D_6_	1688 ± 320	1600 ± 641	2.37*E* − 43	9.44 ± 1.57	9.26 ± 1.95	6.29*E* − 04	1688 ± 320	1600 ± 641	1.33*E* − 57	1835 ± 158	1791 ± 316	1.31*E* − 57
D_7_	1444 ± 260	1393 ± 463	5.14*E* − 39	9.47 ± 1.53	9.27 ± 1.87	1.71*E* − 02	1444 ± 260	1393 ± 463	2.28*E* − 53	1547 ± 128	1522 ± 229	2.34*E* − 53
D_8_	1233 ± 199	1225 ± 291	5.81*E* − 49	9.41 ± 1.45	9.33 ± 1.71	3.00*E* − 06	1233 ± 199	1225 ± 291	4.09*E* − 63	1303 ± 98	1300 ± 143	4.01*E* − 63
D_9_	1033 ± 177	1018 ± 253	3.94*E* − 40	9.35 ± 1.47	9.17 ± 1.74	8.44*E* − 03	1033 ± 177	1018 ± 253	8.76*E* − 53	1089 ± 87	1082 ± 125	7.62*E* − 53
D_10_	864 ± 158	823 ± 262	6.62*E* − 26	9.27 ± 1.51	8.95 ± 1.88	8.40*E* − 03	864 ± 158	823 ± 262	7.05*E* − 35	909 ± 78	889 ± 129	7.39*E* − 35
D_11_	723 ± 129	696 ± 202	1.63*E* − 31	9.17 ± 1.53	8.89 ± 1.85	2.71*E* − 03	723 ± 129	696 ± 202	3.25*E* − 36	759 ± 63	746 ± 100	3.73*E* − 36
D_12_	606 ± 102	591 ± 156	3.00*E* − 46	9.05 ± 1.53	8.86 ± 1.82	3.99*E* − 04	606 ± 102	591 ± 156	2.41*E* − 48	634 ± 50	626 ± 77	1.96*E* − 48
D_13_	509 ± 81	500 ± 123	4.87*E* − 54	8.94 ± 1.53	8.80 ± 1.80	4.07*E* − 06	509 ± 81	500 ± 123	1.13*E* − 52	530 ± 40	526 ± 61	1.56*E* − 52
D_14_	425 ± 64	421 ± 98	3.87*E* − 61	8.76 ± 1.54	8.73 ± 1.79	2.14*E* − 10	425 ± 64	421 ± 98	4.29*E* − 60	442 ± 32	440 ± 48	9.94*E* − 60
D_15_	354 ± 53	352 ± 79	7.96*E* − 64	8.55 ± 1.54	8.62 ± 1.78	2.13*E* − 16	354 ± 53	352 ± 79	7.20*E* − 58	368 ± 26	365 ± 39	1.03*E* − 57
D_16_	296 ± 44	293 ± 67	6.93*E* − 48	8.38 ± 1.53	8.43 ± 1.77	6.72*E* − 14	296 ± 44	293 ± 67	1.26*E* − 42	308 ± 22	306 ± 33	1.33*E* − 42
D_17_	248 ± 35	245 ± 54	1.43*E* − 28	8.24 ± 1.51	8.24 ± 1.75	1.00*E* − 07	248 ± 35	245 ± 54	2.57*E* − 27	257 ± 17	255 ± 27	1.53*E* − 27
D_18_	209 ± 27	206 ± 40	5.19*E* − 16	8.16 ± 1.47	8.16 ± 1.71	5.63*E* − 05	209 ± 27	206 ± 40	1.38*E* − 13	215 ± 13	214 ± 20	1.09*E* − 13
D_19_	176 ± 21	171 ± 35	2.28*E* − 04	8.02 ± 1.42	7.92 ± 1.74	1.05*E* − 03	176 ± 21	171 ± 35	2.40*E* − 03	180 ± 10	178 ± 17	2.47*E* − 03
D_20_	147 ± 17	138 ± 35	4.21*E* − 05	7.82 ± 1.38	7.47 ± 1.79	1.70*E* − 06	147 ± 17	138 ± 35	7.18*E* − 04	150 ± 8	146 ± 17	4.87*E* − 04
D_21_	124 ± 14	114 ± 31	1.73*E* − 31	7.67 ± 1.39	7.08 ± 1.79	5.77*E* − 33	124 ± 14	114 ± 31	2.94*E* − 24	126 ± 7	121 ± 15	9.59*E* − 25
D_22_	103 ± 12	94 ± 27	2.50*E* − 61	7.43 ± 1.41	6.70 ± 1.77	2.55*E* − 59	103 ± 12	94 ± 27	6.44*E* − 48	105 ± 6	101 ± 13	1.61*E* − 48
D_23_	84 ± 11	76 ± 24	1.30*E* − 68	7.06 ± 1.40	6.32 ± 1.77	2.06*E* − 66	84 ± 11	76 ± 24	4.23*E* − 48	86 ± 5	82 ± 12	4.41*E* − 49
D_24_	71 ± 10	64 ± 20	2.10*E* − 82	6.86 ± 1.40	6.08 ± 1.77	5.26*E* − 76	71 ± 10	64 ± 20	6.90*E* − 63	73 ± 5	69 ± 10	4.80*E* − 62
D_25_	57 ± 9	51 ± 17	7.21*E* − 84	6.45 ± 1.43	5.68 ± 1.78	1.00*E* − 76	57 ± 9	51 ± 17	5.41*E* − 63	60 ± 5	56 ± 9	1.47*E* − 62
D_26_	48 ± 9	42 ± 15	7.87*E* − 79	6.16 ± 1.49	5.42 ± 1.81	4.54*E* − 68	48 ± 9	42 ± 15	2.24*E* − 61	50 ± 4	47 ± 8	1.46*E* − 61
A_26_	80 ± 13	74 ± 22	4.93*E* − 44	6.80 ± 1.48	6.25 ± 1.79	1.43*E* − 39	80 ± 13	74 ± 22	4.16*E* − 34	83 ± 6	80 ± 11	1.63*E* − 34

**Table 2:** Performance of classifiers for all entropy-based features.

	KNN	SVM	FFNN	CFNN	GRNN	RNN
ACC (%)	92.44	89.74	93.88	94.77	90.72	93.62
SEN (%)	95.21	93.17	92.92	93.61	89.55	92.36
SPE (%)	89.68	86.32	94.87	96	91.95	94.96

**Table 3:** Performance of classifiers for selected entropy-based features by the BBA algorithm.

	KNN	SVM	FFNN	CFNN	GRNN	RNN
ACC (%)	84.58	82.34	90.62	90.54	79.32	90.18
SEN (%)	85.7	84.34	89.03	88.93	79.46	89.06
SPE (%)	83.46	80.34	92.35	92.29	79.17	91.37

**Table 4:** Performance of classifiers for selected entropy-based features by the BDE algorithm.

	KNN	SVM	FFNN	CFNN	GRNN	RNN
ACC (%)	93.28	89.80	93.12	93.81	91.88	93.69
SEN (%)	95.41	92.85	91.73	92.54	90.67	92.65
SPE (%)	91.14	86.74	94.59	95.16	93.15	94.78

**Table 5:** Performance of classifiers for selected entropy-based features by FA algorithm.

	KNN	SVM	FFNN	CFNN	GRNN	RNN
ACC (%)	92.94	87.98	93.02	92.66	91.42	90.28
SEN (%)	94.96	91.17	92.38	92.05	90.61	88.92
SPE (%)	90.93	84.8	93.69	93.16	92.27	91.73

**Table 6:** Performance of classifiers for selected entropy-based features by GA.

	KNN	SVM	FFNN	CFNN	GRNN	RNN
ACC (%)	93.33	88.14	91.42	93.53	92.21	92.93
SEN (%)	94.93	92.53	90.69	92.59	91.35	91.49
SPE (%)	91.73	83.76	92.18	94.51	93.11	94.47

**Table 7:** Performance of classifiers for selected entropy-based features by the GWO algorithm.

	KNN	SVM	FFNN	CFNN	GRNN	RNN
ACC (%)	93.38	89.41	93.06	93.45	92.06	93.26
SEN (%)	95.54	91.01	92.43	91.66	90.87	92.19
SPE (%)	91.22	87.78	93.71	95.41	93.32	94.39

**Table 8:** Performance of classifiers for selected entropy-based features by PSO algorithm.

	KNN	SVM	FFNN	CFNN	GRNN	RNN
ACC (%)	96.18	92.41	95.48	97.68	95.89	93.59
SEN (%)	98.68	94.08	94.31	97.26	94.93	94.25
SPE (%)	93.69	90.74	96.71	98.11	96.89	94.95

**Table 9:** Comparison of the achieved accuracies among different methods on the same database.

Ref.	Number of EEG signals	ACC (%)	SEN (%)	SPE (%)
[6]	50	90	91.30	91.30
	3750	89.4	88.10	90.7
[10]	50	84	Not reported	Not reported
	750	75		
[15]	50	85	Not reported	Not reported
[16]	50	87	90	84
[17]	50	89	Not reported	Not reported
[18]	50	86	Not reported	Not reported
[19]	50	84	84	84
[20]	3750	83.07	83.5	83.09
[14]	3750	89.52	Not reported	Not reported
[22]	50	90	88	92
	750	82.53	81.60	83.46
[11]	3750	87.93	89.97	85.89
[12]	3750	92.15	94.56	89.74
[13]	50	92.18	92.50	92.69
[33]	3750	84.67	83.86	85.46
[34]	3750	95	Not reported	Not reported
[32]	3750	88.14	Not reported	Not reported
[23]	50	93	100	86
[30]	750	96	94.69	93.50
[31]	3750	95.20	96.10	94.40
[25]	3750	94.41	93.25	95.57
[26]	3750	94.80	92.27	96.10
[24]	50	93	90	90
	3750	82.60	82.60	79.80
[27]	3750	100	100	100
[21]	3750	99.94	99.94	99.94
[29]	3750	99.11	98.52	99.70
[28]	3750	95.58	95.47	96.24
Our method	3750	97.68	97.26	98.11

## Data Availability

No data were used to support this study.
